# General Industrial Environment and Health Design Software Using a Small Data-Driven Neural Network Model

**DOI:** 10.1155/2022/1768446

**Published:** 2022-07-13

**Authors:** Lijun Xu, Jing Zheng, Jun Gao, Wei Chen, Lu Chen

**Affiliations:** ^1^Institute of Art and Design, Nanjing Institute of Technology, Nanjing 211167, Jiangsu, China; ^2^ABB Beijing Drive System Co., Ltd, Beijing, China

## Abstract

The developed enterprise intellectual brain neural network platform for industrial environment and health design driven by small data converts the wisdom knowledge of enterprise designers into data and helps enterprises retain design experience, accumulate design knowledge results, sort out the design process, and shorten the design cycle. The goal of this project is to combine artificial intelligence, big data, the Internet of things, parameterization, and other computer technologies with the industrial environment and health design and development process of manufacturing enterprises to solve pain points for businesses and designers, as well as to develop and create a large-scale product-level general parameter intelligent design software. The development of this software project can greatly improve the work efficiency of designers, save the time spent by designers on low-end repetitive labor, and in turn promote designers to engage in more valuable creative work and realize the digitization of entire product life cycle. It can also improve the inefficient and redundant work efficiency of designers, and designers can switch between multiple roles. At the same time, a design think tank is formed through the accumulation of enterprise design knowledge through data, and the neural network platform development of big data drives the design brain, that is, an efficient and intelligent industrial environment and health design expert system is generated, just like the enterprise brain, including expert think tanks, internal technical data encryption of enterprises interface, enterprise core technology think tank, enterprise production resources, risk control standard library, etc.

## 1. Introduction

Technological innovation is mainly reflected in the digital transformation of manufacturing industry. The development overview and latest development trends of various aspects are as follows.

Increasing global competition is driving companies to become more economically, environmentally, and socially sustainable. To be truly sustainable, businesses must build truly intelligent systems (both manpower and technology) that can respond quickly and flexibly to changing circumstances. Existing companies cannot survive in the future without improving their digital capabilities. Building a sustainable digital enterprise is the inevitable development of the times.

The people's governments of Jiangsu Province and Nanjing Municipality will work together to fully implement the manufacturing a strong country and digital China development strategy, further implement the work arrangements of the Municipal Party Committee and Municipal Government on accelerating the development of the digital economy, and comprehensively promote the digital transformation and high-quality development of the city's manufacturing industry (2021–2023). These steps will help to accelerate the manufacturing industry's digital transition and build a new engine for high-quality digital economy development. It is suggested that by 2023, the city's manufacturing industry's degree of digitization, networking, and intelligence will be greatly increased, and the digital transformation ratio of industrial companies will reach 70% [1, 2].

The Jiangsu Provincial Department of Industry and Information Technology, the Provincial Department of Science and Technology, and others support industrial environment and health design software technology research, product development, and solution integration, as well as the development of an open source ecosystem for industrial environment and health design software based on enterprise needs for “intelligence and digital transformation.” The first edition of the secondary industrial environment and health design software application promotion guidance catalog was published and more industrial environment and health design software products were promoted to enter the national industrial environment and health design software supply capacity list, thus encouraging manufacturing enterprises to use the software products in the catalog and the list to promote “intelligent and digital transformation” [3]. By the end of 2024, the province's annual revenue from industrial environment and health design software products is expected to exceed 85 billion yuan, with a total of 8 breakthroughs in industrial environment and health design software key core technologies, support for more than 100 industrial software R&D applications, promotion of more than 4,000 industrial APPs, and the formation of 2–3 internationally competitive industrial software well-known brands.

The worldwide industrial intelligence development scale is expanding day by day in the “Industry 4.0” age, and its impact on modern industries cannot be overstated. Traditional industries' innovation skills have been continuously strengthened by technologies such as big data, artificial intelligence, and virtual reality, and the more skills the traditional companies have, the more prospects for future development they will have. In the face of tremendous disruptive developments brought about by emerging technologies, the future development of industrial design has ushered in enormous development potential. The value development of high-tech lies at the heart of “Industry 4.0.” China is both a large producer and a large consumer. In China, a vast amount of data consumption can be acquired. China is likely to reap significant benefits from the “Industry 4.0” wave. China's design sector is facing the possibility for change as a national growth plan, against the backdrop of “Industry 4.0” [4].

Our country is in the era of information explosion, the prosperity of science and technology will make the nation prosper, and the strength of science and technology will make the country strong. The progress of science and technology is important; however, if the progress of science and technology is not implemented in the application of industry, then the value of science and technology will not be reflected. “Industry 4.0” is founded primarily on nine digital industrial technologies, including industrial Internet of things, cloud computing, industrial big data, industrial robotics, 3D printing, virtual reality, and artificial intelligence [5].

Based on independent control, the software development of this project promotes the advanced industrial software industry foundation and iterative upgrading of industrial software solutions and focuses on breakthroughs in R&D design, business management, production scheduling, and process control industrial software, such as EDA software, and basic supporting software, such as operating system and database. It will promote the in-depth application of independent simulation technology in various industries and solve the problem of “stuck neck” in industrial software.

In the age of big data, big data and little data are not diametrically opposed, but rather a unity that depends on one another, and the two play diverse values and roles at their respective levels. Small data does not refer to small-scale data. It refers to a data set with multisource, heterogeneity, dynamics, and holography centered on specific objects, guided by responding to specific needs and aimed at solving specific problems, as well as the thinking mode and data processing method of related data acquisition, processing, analysis, and human-computer interaction [5]. Small data is high-quality data that can be used to support intelligent decision-making in enterprises. Without complex algorithms and expensive costs, any enterprise can realize the analysis and application of small data.

Big data and small data are not opposites, but unity. Small data is an aspect of big data. After collecting, expanding, and linking small data to form a larger data set, small data will become more and more close to big data. The data processing paradigm of information can effectively make up for the defects and deficiencies of big data in dealing with specific scenarios, targeting specific goals, and meeting special needs.

The data values of big data and small data mining have their own advantages. On the one hand, big data mining does not have the potential value of specific data, and small data releases the explicit value of specific data; on the other hand, big data finds laws based on correlation, while small data verifies laws based on causality. Integrating big data and small data can help enterprises solve the problems of digital transformation.

In 2009, Wang Guoxin and others proposed a modeling method combining data-driven and modular control model, which can quickly and accurately provide the data required to create the simulation model, avoiding the errors and low modeling efficiency caused by a large number of human-computer interaction in the traditional modeling methods [6, 7]. The modular modeling method divides the complex model into various independent functional modules, which is convenient for the maintenance and expansion of the model. Through the specific application of this method, it is proved that the combination of data-driven and modular modeling method provides effective technical support for the rapid establishment of simulation models of large and complex systems.

The predicament of big data-driven enterprise transformation is that, first, there is a performance bottleneck in big data analysis and processing; second, there is a disconnect between enterprise big data applications and actual business needs; and third, the level of digital collaborative development among enterprises is not high. To break through this predicament, it is necessary to promote the integration and application of big data and small data. Big data brings unprecedented opportunities for the digital transformation of enterprises, but big data is still in the initial stage of development. Only with the integration and development of small data, the application of big data can be better promoted.

This project lays a foundation for generalized product design through standardized data structure representation, changes the long-standing situation of rapid product design and secondary development and customization, and gets rid of the intricate relationship between software developers who have a comprehensive grasp of all product design processes and data organization and operations; the application of software allows software development and product design to return to the original and give full play to their respective strengths. Product technical agreement data is the product agreement specification description data of each enterprise, which belongs to small data. Driving product design through product technical agreement data, that is, small data, is a small data drive that conforms to the actual situation.

An artificial neural network is a mathematical model that imitates human nerves, and it is an artificial intelligence computing method with real-time learning and knowledge acquisition capabilities [8]. Industrial design is a systematic project, which has the characteristics of multi-indicator and multifactor, and each indicator factor is divided into qualitative and quantitative factors. The weight of the comprehensive evaluation index is closely related to objective reality. The artificial neural network knowledge is used to quantify the index, and each design parameter is defined as a network node. The scheme is designed and optimized based on the general mechanical design principle, which is a technological method of digital and intelligent design.

Product design is a multidisciplinary and highly coupled multistage complex process, which not only includes a large number of computational work based on mathematical models and numerical processing but also involves reasoning and decision-making processes based on symbolic knowledge models and symbolic processing, such as the selection of design options; evaluation, modification, and optimization of main parameters; generation of geometric models; and analysis of computational simulation and other design activities. The completion of these tasks requires not only the help of computer-aided design tools but also the use of a lot of knowledge for reasoning, judgment, and decision-making.

Computer-aided industrial design takes industrial design knowledge as the main body and uses computer network and other information technology as auxiliary tools to realize the real description of products, so as to better design economical and beautiful innovative products to better meet people's needs. Computer-aided industrial design is a product of the computer age. Compared with traditional industrial design, it not only optimizes the method and process of industrial design but also effectively improves the quality and efficiency of design.

Wang Guoxin of the Beijing Institute of Technology presented a knowledge service technique to support the intelligent design of goods, which is a human-computer interaction intelligent design activity carried out with the help of computer-aided design tools by integrating multidomain knowledge [9]. Product design and knowledge reuse can be realized intelligently with the help of knowledge engineering technology and artificial intelligence technology to replace the decision-making and reasoning process of experts and designers by building a knowledge environment oriented to the design process, thereby reducing the cycle iteration time in the product design process and reducing repetitive work.

With more research into the intersection of computer technology and industrial design technology, new technologies such as virtual reality, neural networks, and genetic algorithms, as well as design methods such as concurrent design and aided design, have gradually emerged as another hotspot [10, 11]. The neural network system is more complex. He first conceptualized the information and represented it with computer symbols and then used computer software for reasoning and analysis to form computer instructions and then execute them. The massive information storage and analysis ability of the computer can help industrial designers obtain stronger knowledge support, and the spatial expression ability of computer can help designers express their inner design ideas more accurately.

In the design of series products or nonstandard products, we will collect all-around data of the product design process in order to solve the problem of repeating the design of a large number of parts. We will then use neural network technology to mine the relationships between the data. The reliability of product design and automatic drawing is greatly improved.

China's economic take-off in the past three decades has basically been driven by investment and resource consumption. Most enterprises control economic operations and inflate commercial value by occupying land resources, cheap labor resources, scarce mineral resources, and even political power resources. However, the accelerated exhaustion of old resources has become the reality of design integration and innovation in the era of severe intellectual brains on a global scale—a more rational and intelligent development model has increasingly become the inherent demand of enterprise transformation and social progress.

In 2020, Yu Min proposed that the “enterprise brain” is a shared platform for enterprise data [12]. It realizes data interconnection, sharing, synchronization, analysis, and processing, solves the problem of data islands within the enterprise, and provides a variety of smart applications. It provides a unified data platform and interface to realize the intelligent transformation of enterprises, so as to promote the opportunity of generating profit from virtual assets of data and information and enhance the comprehensive competitiveness and economic benefits of enterprise development.

In 2021, experts such as Giovanni Schiuma pointed out that businesses that gain sustainable competitive advantage in the digital age face the challenge of developing transformative digital leadership marked by a range of capabilities [13]. In the digital age, advancements in technology enable the deployment of new products and services to better enhance a company's productivity and customer demand satisfaction. In addition, digital innovation helps to generate vast amounts of data, information, and knowledge, which, if codified and exploited, may yield valuable insights for companies, aligning decision-making and production outputs with market demands.

Arturo Molina suggests designing and building a business that is aware, intelligent, and sustainable in answer to the difficulties of the digital enterprise. Achieving manufacturing sustainability necessitates a comprehensive approach that includes not just the goods and manufacturing processes involved but also the whole supply chain, including manufacturing systems that span many product life cycles.

Design is the beginning of the operation of an enterprise, and the digitization of design is crucial to the digital transformation of an enterprise. This project develops and builds an enterprise design brain, constructs a digital design knowledge base, carries out digital transformation and informatization upgrade of enterprise design, realizes the intelligent accumulation and application of real-time massive design data, and overcomes the losses caused by the loss of designers to enterprises. It will help the digital transformation and intelligent transformation of enterprises and create a model of the whole industry chain design of smart factories.

The project is oriented to industrial design. Through the data neural network architecture environment, small data drives the enterprise brain, carries out innovative intelligent design, and realizes the digitization of the wisdom of enterprise designers. It will help enterprises retain design experience, accumulate design knowledge achievements, sort out the design process, and shorten the design cycle. The creation of design smart brain belongs to the top-level architecture of enterprise digital transformation. In order to realize the intelligent manufacturing of the whole product life cycle, the smart brain formed by the software application, as the beginning of enterprise intelligent manufacturing, will help the whole cycle digital transformation of manufacturing enterprises.

## 2. Research on the Function and Value of General Industrial Design Software

### 2.1. Definition and Methods of Industrial Design

In 2015, the International Society for Industrial Design (ICSID) held its 29th Annual Congress in South Korea. The acronym “ICSID,” which has been in use for nearly 60 years, will be formally renamed “World Design Organization” and defined as follows [14]: Industrial design is a design activity that applies a strategic problem-solving method to goods, systems, services, and experiences in order to guide innovation, promote commercial success, and improve quality of life. It is an interdisciplinary profession that closely connects innovation, technology, business, research, and consumers to jointly engage in creative activities such as visualizing problems to be solved, proposing solutions, and re-deconstructing problems; and it serves as an opportunity to build better products, systems, services, experiences, or business networks, providing new value and competitive advantage. Through its output, industrial design responds to social, economic, environmental, and ethical challenges with the goal of creating a better world. The definition here clearly recognizes the upgrading of industrial design definition, the expansion of orientation, and the emergence of the pattern. The design of the industrialization and information age, the harmonious design of living, and the new shape of current culture are all examples of industrial design.

*Computer-Aided Industrial Design Methods*. The development of computer technology and network technology provides new media and tools for modern design methods and plays an important role in modern industrial design. Most product designs are inseparable from the support of computer technology. With the increasing maturity of computer software and hardware and the continuous development of CAD/CAM technology, computer-aided industrial design (CAID) technology has become a research hotspot in the fields of industrial design and advanced manufacturing [6]. CAID's mission is to perform various creative activities in the field of industrial design with the assistance of computers and their associated software systems [6]. The use of CAID technology can significantly improve the product's overall design quality.

At present, the research on CAID technology at home and abroad mainly focuses on auxiliary modeling technology (NURBS surface design, modeling parametric design, sketch design, etc.), human-computer interaction technology (human-computer interface technology, virtual simulation technology, etc.), intelligent technology (intelligent CAD, intelligent design), high-tech (virtual reality, neural network, genetic algorithm, concurrent design, collaborative design, VR-based product design), and other aspects [15–17]. Industrial design modules [10, 18–20] are provided in some engineering design software (such as UG, CATIA, EDS, and Unigraphics), which provides a platform for the coordination of industrial design and engineering technology [6]

To summarize, in modern industrial design, designers who rely on tacit knowledge, experience, and qualitative judgment cannot meet the needs of design needs and the design process, and the development trend of industrial design methodology is to adopt scientific, quantitative, and accurate research methods. Multidisciplinary collaborative and cross research has become the main method of industrial design, drawing on natural science research methods, modern scientific and technological achievements, and relevant humanities knowledge. According to some academics, modern industrial design is a system engineering design [10].

### 2.2. Overview of General Industrial Design Software

The application of industrial intelligent design software can improve the R&D and design ability of enterprises. The product design knowledge and experience can be self-recorded and integrated in the whole process, so as to realize data integrated management. Designers can spend limited time on more valuable creative R&D work and free themselves from redundant low-end labor. The standardized data structure expression lays the foundation for generalized product design, changes the long-standing situation of rapid product design and secondary development and customization, and gets rid of the intricate relationship between software developers who have a comprehensive grasp of all product design processes and data organization and operations. The application of software allows software development and product design to return to the original, giving full play to their respective strengths.

1. The smallest unit of the model is noded, the product structure is networked, and data are used to build products; the rules of drawing are expressed in language, and data are used to create two-dimensional drawings in real time; and the digitalization of the design process can accelerate the digital transformation of enterprises.
2. Every detail is recorded in the whole process, which is easy for the inheritance and self-learning of design knowledge and improves the ability of enterprise design and development technology iteration.
3. The creation of a design think tank belongs to the top-level structure of an enterprise's digital transformation. To realize intelligent manufacturing in the full life cycle of a product, the think tank formed by this software application, as the beginning of enterprise intelligent manufacturing, will help manufacturing enterprises in their full-cycle digital transformation.

The purpose is to solve the problems of repetitive product design, such as serial design or nonstandard design. The project has conducted all-round data research and exploration on the product design process, process, method, data, model, drawing, and BOM and established a complete set of small data-driven neural network data high-end general intelligent design software. The description system and expression method of product design data are established, which can be copied, repeated, and maintained. Engineers build the neural network architecture environment of product design data by themselves, which greatly improves the reliability of product design and automatic drawing.

## 3. Research Content of General Industrial Design Software

The neural network data architecture driven by small data can fully adapt to the extraction of model data, the evolution of model data, and the composition of assembly. Similarly, the neural network data architecture driven by small data shows its adaptability, controllability, and adjustability in drawing generation. This project focuses on the neural network data architecture driven by small data and the control of drawing generation technology and puts forward the concept, application and implementation, and control the application points of technology, so as to make all functions of the software meet the envisaged requirements and ensure the implementation of the project. The neural network data architecture and drawing technology driven by small data lay the foundation for the implementation of the project.

### 3.1. Research and Design of the Neural Network Architecture Environment Environment of Data Generated by Industrial Products in Digital Transformation and Realizing Small Data-Driven Innovative Design

We analyze the traditional design process of enterprises; face the digital transformation of design, study the effective protocol data, total product design parameter data, size data, etc., of the driven design, study how to establish the association between discrete data, establish design rules, and form the neural network structure of the data; through the analysis and research of data and the construction of association rules, we realize the innovative design of products based on small data.

### 3.2. Research on Small Data and Data-Driven Engine Technology of Product Design in the Industrial Design Process

The general data architecture is established for small data-driven neural network data, which proves its feasibility and practicability. In terms of architecture research, how to improve and expand the data, improve the adaptability and maintainability, fully meet the whole process data flow of product design requirements, and prove that the data architecture is universal and reasonable? In terms of software framework, software data has reliability, customization, expansibility, scalability, and maintainability. Because it adopts the form of Excel database, it has these functions. Excel establishes data expression and data specification. Of course, the selection of interface software design software for mainstream design products of industrial products also improves the requirements of openness and data maintainability of 3D model data, paving the way for data to 3D model display. At the same time, the leading degree of drawing technology determines the effect that can be realized. The program here only realizes the function and data association and plays a great role. The automatic control of the transmission between the total design parameters and the model design table and the display of automatic design and automatic generation of two-dimensional drawings need to be improved and implemented by the software one by one. The architecture diagram of small data-driven neural network is shown in Figure 1.

### 3.3. Using Computer-Aided Industrial Design Methods to Realize 3D Digital Modeling and Automatic Generation and Optimization of Products

The original design software has an all-round control function for the three-dimensional model. We can use the API interface function to control the sketch size on the three-dimensional model, model feature control, feature data compression, position adjustment of the assembly, reinstallation of the assembly model, control the presence or absence of the model in the assembly, etc. In the process of product evolution, the final requirements of product design are fully met.

The product design displayed in the computer is generally 3D model design software. Currently, the commonly used 3D design software includes UG, ProE, interface software for mainstream design products of industrial products, etc. Taking the interface software of the most widely used mainstream design products of industrial products as an example, the correlation between the model size and the total design parameters of the product is illustrated from the data point of view. Automatically optimize 3D design model drawings are shown in Figure 2.

### 3.4. Using Small Data-Driven Engine Technology to Automate the Design of Large and Complex Machines for Industrial Products

The small data-driven neural network data can design any combination of nonstandard products within the rules, providing an imaginary space for the company's subsequent product design. As long as there is a 3D model and the corresponding model control parameter description, the 3D automatic assembly and design automation of the large and complex complete machine of industrial products can be realized.

### 3.5. Using Neural Network Architecture Environment to Automatically Generate 2D Engineering Drawings of Industrial Products in Real Time

The general data architecture proves its feasibility and practicability for the establishment of small data-driven neural network data. Automatically control the transfer between the total design parameters and the model design table and the display of automatic design and automatic generation of two-dimensional drawings will be realized one by one.

The storage of design data in the neural network needs to consider the openness of the data and the convenience of self-maintenance. Users can adjust and update the data at any time. According to the above-mentioned contents, product design data are of various types, huge amount of data, and complicated. The use of conventional databases has poor openness, and its calculation formulas cannot be implemented one by one. The calculation formulas in the database are difficult to express, and personnel with rich database development language experience are required. The application threshold is high, which is not conducive to promotion. In the current project, the most commonly used Excel database is used, and the specific openness, compatibility, self-maintenance and adjustment at any time, various size calculation formulas, and logical judgment processing can be realized. As long as the project formulates data filling rules, regional rules, various writing expressions, etc., and the fill-in person fills in the specified area according to the rules and forms, it can meet the basic needs of the data. In terms of software, error proofing of data is also considered. We build product design data in the EXCEL platform, allow users to build the Neural Network Architecture Environment Environment of product design data, make product design demand data easy to standardize, guide users to fill in standard data, and train companies to understand product development from the perspective of mathematical modeling. The amount of product design data is huge and complicated. How to construct neural network data and how to associate these neural network data require certain teaching and training so that users can gradually master the standardization and correct expression of data representation. The neural network data atlas is shown in Figure 3

## 4. Application Research of Enterprise Intelligent Brain Industrial Design Software

### 4.1. Research and Development of Neural Network Platform for Small Data-Driven Design of Intelligent Brain

The research and development of the neural network platform can enhance the innovation ability of enterprises and the creativity of designers' business, increase the replicability of successful experience models and methods, clarify the logic of the design process, and effectively correlate various discrete data with the original design program:

1. After the project requirements are put forward, the designer needs to analyze, classify, organize, and correct a number of data; by sorting and rating the validity, fault tolerance, and efficiency of the project data, the value prediction of the project can be obtained.
2. Designers search for data standards by benchmarking, convert project planning data into underlying parametric software data, set parameters accordingly, and build a 3D parametric model.
3. Designers ensure the correctness of data nodes through data research and judgment, manually participate in the evaluation of the settings of the underlying complex parameters, and control key quality and risks.
4. Designers inefficiently and redundantly engineer the underlying data and convert 3D parametric models into technical documents that can be executed by various departments. Designers need to switch between multiple roles, which hinders the overall work efficiency of each department.

The designer's design pain point process is shown in Figure 4.

### 4.2. The Design of Intelligent Brain

The research and development of the neural network platform can set up an efficient intelligent engineering design expert system, which is like an enterprise brain. It includes expert think tank, internal technical data encryption interface, enterprise core technology think tank, enterprise production resources, and risk control standard library. The details are as follows:

1. After the project is proposed, the expert think tank instructs the designer to sort out the demand data of the project and sort out the effective agreement data.
2. The internal technical data encryption interface of the enterprise can efficiently transform the underlying parameters of the effective protocol data input by the designer, which can not only ensure the circulation of external protocol data but also isolate the leakage of internal core algorithms; then carry out the monotonous cycle of the enterprise's core technology think tank, control the enterprise's production resources and risks, and efficiently implement and copy the standard library to quickly convey the technical documents of various departments.
3. The core technology think tank of the enterprise includes data bottom parameterization, construction of three-dimensional parameter model, and data evaluation.
4. The standard library of enterprise production resources and risk control includes converting the underlying data engineering and 3D parametric models into technical documents executable by each project department upstream and downstream resource libraries, multidata type conversion algorithms, logical models, and multidata input and output interfaces.
5. The results are evaluated by both artificial and virtual simulation, and the experience of the project design results is summarized.
6. Transmit the technical documents of external output to each corresponding executive department, thus promoting the growth of the enterprise's brain system.

The process of designing the brain is shown in Figure 5.

### 4.3. Taking the Enterprise Brain as the External Resource of the System Can Make the System More Universal

The high-end general industrial design software driven by enterprise intelligent brain based on neural network architecture environment is an intelligent software platform for smooth transmission, operation, and execution of multiple data types. At the same time, the wide interface of the platform provides a high-speed channel for input and output of multiple types of data. Connecting with the enterprise intelligent brain guiding the execution of the software can effectively and organically correlate a large amount of discrete underlying parameters, learn the experience after each successful project, and internalize the data and accumulate enterprise knowledge database to promote the growth of enterprise intelligence. At the same time, transmitting intelligent brain information through data interface can also improve the information security of intelligent brain. The enterprise brain process is shown in Figure 6.

1. After the project is proposed, the designers sort out the project and design a small amount of valid agreement data related to the project.
2. Valid protocol data enters the system, the project experts owned by the enterprise intelligence brain explain the think tank, the internal core technology data model library of the enterprise guides the system to perform algorithm matching on the multidimensional protocol data, reduce the test protocol data to the underlying basic parameters, and build the basic parameter model of the project; under the guidance of the brain of the enterprise, the system conducts data research and judgment on the test parameter model. If the agreement data is wrong, it will feed back to the external designer to reconfirm and modify the agreement data. If the agreement data passes the research and judgment, the algorithm will be iterated. Optimize the parameters until the parameter model is qualified.
3. In this process, through the dimensionality reduction of protocol data, a large amount of discrete bottom parameterized data can be formed. Through the intelligent brain algorithm and the parameterized model required by the model test project, the algorithm can be iterated and optimized until it is qualified through internal research.
4. The parameter model performs a fully enclosed hidden test inside the system and feeds back the test data. Under the guidance of the enterprise intelligence, the parameters or parameter associations associated with the test unqualified indicators are corrected until all the indicators in the simulation test are qualified.
5. Under the guidance of the enterprise's brain, the system performs multiple data translations and transfers for qualified parameter models to form technical documents required by each project execution department.
6. The system translates and outputs the underlying parameter model to the outside. Designers can summarize design experience through visual external data results. Machines can learn from the data and internalize them into the corresponding think tank data and algorithms in the enterprise brain. Algorithms continue to accumulate, promoting the growth of corporate intelligence.

### 4.4. Enterprise Brain and Smart Factory Are Synergistic, Complementary, and Mutually Reinforcing

The enterprise brain is made up of the enterprise think tank and the digital twin factory. The enterprise think tank can be divided into six different types, including production and operation strategy base, project execution rule base, core technology logic base, internal data transfer rule base, enterprise resource management logic base, and overall risk control strategy base. Six different types of database are independent and related to each other, which together constitutes the enterprise think tank. The enterprise think tank guides the digital twin factory in terms of control, logic, judgment, and decision-making.

The digital twin factory is a virtual mapping of the real smart factory, which plays the role of overall planning, intelligent control, and rational operation of the real smart factory. The real smart factory needs to give full play to its physical functions, relying on big data technology to perform extensive calculations, comprehensively debug and optimize the design scheme, and finally complete intelligent design, accurately control intelligent production, and efficiently implement intelligent decision-making.

In turn, the real smart factory verified by practice will also “feed” its digital twin factory, play the role of experience guidance, constantly enrich the enterprise think tank in the four aspects—control, logic, judgment, and decision-making—and finally make the enterprise brain more intelligent, forming a closed loop. Details of the synergy between the enterprise brain and the smart factory are shown in Figure 7.

1. Expanding the intelligent design module in depth. When the real smart factory receives a project task, the intelligent design module first checks the project agreement data effectively and efficiently builds a technical rule data model, then judges the technical rule data model, checks the standard and compares it to the best, and continuously optimizes it.
2. The project rule data model controls the underlying parametric model building system. The intelligent design module will first parameterize the underlying data, then use the parameterized underlying data to build a three-dimensional parametric model, judge and adjust the three-dimensional parametric model monotonically and error-free, and ultimately achieve the purpose of continuous optimization.
3. Multidirectional translation of the underlying parametric model allows for the engineering of the underlying data, which transforms the 3D parametric model into technical documents that can be implemented by various project departments. These technical documents can be efficiently replicated, which facilitates the summation of experience and facilitates machine learning of relevant data, internalizing the data and ultimately supplementing and updating the knowledge of the enterprise brain, which is constantly being improved.

## 5. Conclusions and Prospects

The innovation of this project lies in the use of small data-driven technology for the first time in the process of product innovation and design; through the standardization of product design data description, the universal use of software in all fields can be realized; with the help of neural network architecture environment, the closed-loop optimal design of industrial products is realized.

A complete set of neural network data organization system driven by small data is built and expressed through universal and standardized format data. The corresponding software processing program has been compiled to make the vision come true. The software solves the automatic construction and assembly process of the minimum unit three-dimensional model, which makes the mathematical modeling and assembly possible. The data evolution and data combination can produce a new assembly model body completely according to the customized rules, so that the mathematical description and mathematical combination can be synchronized and consistent with the three-dimensional model assembly. Deepen the application of product mathematical modeling, and let everyone master the method of product mathematical modeling. Master the leading technology of drawings, make drawings into real-time generation, make the generation of drawings digitized and logical, and standardize the description of data. Changes in drawing data make the evolution of drawings digitized, controllable, and automated. Let the original model correspond to a drawing control form, and generate a large number of evolution models and corresponding drawing methods, which are fully digitized and characterized.

The original drawing data is the final result of enterprise control, but now it is changed to comprehensive control process, process, method, calculation, judgment, etc., and the data is recorded in the whole process. It will provide complete data for enterprises to build product design knowledge bases and comprehensive data documents for product design knowledge inheritance and product data iteration.

## Figures and Tables

**Figure 1:** Architecture diagram of small data-driven neural network.

**Figure 2:** Automatically optimize 3D design model drawings.

**Figure 3:** Neural network data atlas.

**Figure 4:** Designer's design pain point process.

**Figure 5:** The process of designing the brain.

**Figure 6:** Enterprise brain process.

**Figure 7:** Details of the synergy between the enterprise brain and the smart factory.

## Data Availability

The data set used to support the findings of this study is available from the corresponding author upon request.
